The article "Machine Learning-Based Prediction of COVID-19 Prognosis Using Clinical and Hematologic Data" was retracted in 2026. Reasons: unreliable results or conclusions; concerns about the data; concerns about the methods; concerns about the results or conclusions.

# Machine Learning-Based Prediction of COVID-19 Prognosis Using Clinical and Hematologic Data

**DOI:** 10.7759/cureus.50212

**Published:** 2023-12-09

**Authors:** Fatemah O Kamel, Rania Magadmi, Sulafah Qutub, Maha Badawi, Mazen Badawi, Tariq A Madani, Areej Alhothali, Ehab A Abozinadah, Duaa M Bakhshwin, Maha H Jamal, Abdulhadi S Burzangi, Mohammed Bazuhair, Hussamaldin Alqutub, Abdulaziz Alqutub, Sameera M Felemban, Fatin Al-Sayes, Soheir Adam

**Affiliations:** 1 Department of Clinical Pharmacology, King Abdulaziz University Faculty of Medicine, Jeddah, SAU; 2 Preventive Medicine, College of Medicine, Jeddah University, Jeddah, SAU; 3 Department of Hematology, King Abdulaziz University Faculty of Medicine, Jeddah, SAU; 4 Section of Infectious Diseases, Department of Medicine, King Faisal Specialist Hospital and Research Centre, Jeddah, SAU; 5 Department of Medicine, King Abdulaziz University Faculty of Medicine, Jeddah, SAU; 6 Department of Computer Science, Faculty of Computing and Information Technology, King Abdulaziz University, Jeddah, SAU; 7 Department of Information Systems, Faculty of Computing and Information Technology, King Abdulaziz University, Jeddah, SAU; 8 Intensive Care Unit, King Fahad General Hospital, Jeddah, SAU; 9 Hematology Section, Medical Department, King Fahad General Hospital, Jeddah, SAU; 10 Department of Medicine, Faculty of Medicine, Duke University, Durham, USA

**Keywords:** prognosis, hematology, clinical prediction, covid-19, artificial intelligence

## Abstract

The coronavirus disease 2019 (COVID-19) pandemic is challenging healthcare systems worldwide. The prediction of disease prognosis has a critical role in confronting the burden of COVID-19. We aimed to investigate the feasibility of predicting COVID-19 patient outcomes and disease severity based on clinical and hematological parameters using machine learning techniques. This multicenter retrospective study analyzed records of 485 patients with COVID-19, including demographic information, symptoms, hematological variables, treatment information, and clinical outcomes. Different machine learning approaches, including random forest, multilayer perceptron, and support vector machine, were examined in this study. All models showed a comparable performance, yielding the best area under the curve of 0.96, in predicting the severity of disease and clinical outcome. We also identified the most relevant features in predicting COVID-19 patient outcomes, and we concluded that hematological parameters (neutrophils, lymphocytes, D-dimer, and monocytes) are the most predictive features of severity and patient outcome.

## Introduction

The current coronavirus disease (COVID-19) pandemic has strained the healthcare systems worldwide. Within 18 months of the start of the pandemic, there were more than 185 million confirmed cases and four million deaths worldwide [1]. The availability of medical resources plays a significant role in the variation in death rates among countries [2]. In many places, the demand for intensive care units (ICUs) exceeds the capacity of facilities. Therefore, it is critical to take a proactive approach to utilizing healthcare resources, such as ICUs, to maintain healthcare delivery throughout the COVID-19 pandemic. Consequently, predicting the prognosis of patients with COVID-19 (outcome and severity) as early as the time of admission can help provide clinical care and effectively utilize medical resources. Researchers have identified several indicators that aid in COVID-19 diagnosis and prognosis. For example, cough, fever, chest pain, and dyspnea are common symptoms experienced at the beginning of a viral infection [3]. Moreover, previous studies have found that hematological and biochemical parameters indicate COVID-19 disease [4-6]. However, machine learning can be used to predict the prognosis of many diseases based on clinical and hematological data [7,8]. This study explored the feasibility of predicting COVID-19 patient outcomes and disease severity based on clinical and hematological parameters using machine learning techniques.

The article "Machine Learning-Based Prediction of COVID-19 Prognosis Using Clinical and Hematologic Data" was retracted in 2026. Reasons: unreliable results or conclusions; concerns about the data; concerns about the methods; concerns about the results or conclusions.

Recent studies have investigated machine learning methods trained on COVID-19 patient data to predict their prognosis [9,10]. Researchers examined patient information acquired during admission, including patients’ initial physical examination results and blood count test results, to diagnose patients or predict the severity of the disease. However, the current study examined several machine learning models to predict patient outcomes (i.e., death/recovery) and disease severity (i.e., discharge or admission to ICU). We also investigated the most influential features, such as demographic data, and symptoms at admission, such as fever, cough, sore throat, loss of smell and taste, and gastrointestinal disturbance, that can aid in the prediction of COVID-19 patient outcomes and severity. In addition, this study examined a different set of features, such as medical treatments and comorbidities that have not been previously studied.

## Materials and methods

Data and patient cohort

This was a multicenter retrospective study. Participants’ data were extracted from patients’ electronic files from three main governmental hospitals in Jeddah, Saudi Arabia (King Abdulaziz University Hospital (KAUH), King Fahad General Hospital, and King Abdullah Medical Complex). Patients who were aged 18 years and older and admitted with positive COVID-19 polymerase chain reaction (PCR) results during the peak of the COVID-19 pandemic (March-May 2020) were included in the study. All participants with negative COVID-19 PCR results and those aged <18 years were excluded. The study protocol was approved by the Bioethics Committee at KAUH (Reference No. 271-20) and the Ministry of Health (MOH) (20-87E). Each patient’s record had 48 numerical and categorical attributes, including demographic information, comorbidities, symptomatic observations, hematological variables, medical treatments, and outcomes.

The article "Machine Learning-Based Prediction of COVID-19 Prognosis Using Clinical and Hematologic Data" was retracted in 2026. Reasons: unreliable results or conclusions; concerns about the data; concerns about the methods; concerns about the results or conclusions.

The demographic data included age, sex, nationality, and job (whether working in the healthcare domain or not). The comorbidities considered in this study were diabetes mellitus, hypertension, respiratory, malignancy, and cardiovascular diseases. The clinical data examined in this study consisted of eight categorical features/attributes that were acquired from patients’ initial evaluation at admission, including temperature/fever, dyspnea, sore throat, cough, loss of smell and taste, and gastrointestinal disturbance, such as diarrhea and vomiting. The hematological variables consisted of 21 numerical variables, including hemoglobin level (HL), red blood cells (RBC), white blood cells (WBCs), basophils, neutrophils, monocytes, lymphocytes, eosinophils, and D-dimer. Patient information also comprises the prescribed medications given during the treatment plan, including paracetamol; anticoagulants; antibiotics, such as azithromycin; antiviral agents, such as oseltamivir; Kaletra, which is a combination of two lopinavir and ritonavir; and hydroxychloroquine.

Data pre-processing

To compensate for missing values in the dataset, we examined two strategies. First, we imputed missing numerical values with the attribute mean value and missing categorical values with the most frequent category if the missing values do not exceed 10. To transform categorical data into numerical data, we employed a transformation technique to encode label categories (e.g., Yes and No) into their numerical representation. We also applied a standardization technique (Z-score) to scale the range of input dataset to reduce the significant difference between the minimum and maximum values and reduce the difference between attributes measured in different measurement units. The dataset was imbalanced in that it has an unequal class distribution: 386 cases of recovery and 99 deaths, 371 not admitted to the ICU, and 114 admitted to the ICU. Class imbalance is a challenging problem in predictive modeling. This dataset is considered mildly imbalanced, as the minority class contributes 20-23% of the entire dataset. To handle this class imbalance, we used a stratified sampling technique to divide the dataset into training and test sets.

The article "Machine Learning-Based Prediction of COVID-19 Prognosis Using Clinical and Hematologic Data" was retracted in 2026. Reasons: unreliable results or conclusions; concerns about the data; concerns about the methods; concerns about the results or conclusions.

Machine learning models

We implemented several machine learning algorithms to predict the clinical outcomes (i.e., death or recovery) and complications of patients with COVID-19 (i.e., the need for ICU admission). Specifically, we used logistic regression (LR), multilayer perceptron (MLP), random forest (RF), support vector machine (SVM), naive Bayes (NB), and extreme gradient boosting (XGboost). Each of these standard models belongs to a different family of machine learning models: tree-based models for RF, linear models for LR and SVM, probabilistic models for NB, and ensemble learning for XGboost. We applied a hyperparameter optimization technique to select hyperparameters that provide optimal accuracy. For LR, the optimal results were obtained using C, regularization penalty, and compiler/solver equal to 0.55, L1, and liblinear, respectively. For MLP, the optimal learning rate, activation function, alpha, hidden layer sizes, and solver were adaptive, tanh, 0.0001, (50, 50, 50), and sgd, respectively.

For the SVM, the hyperparameters C, gamma, and kernel are equal to 10, 0.001, and rbf, respectively. For the NB algorithm, the optimal smoothing variable was set to 1.0. For XGboost, the learning rate, maximum depth, and minimum child weight were 0.01, 3, and 3, respectively. For the RF, the splitting criterion is entropy, the maximum depth is equal to six, and the maximum number of features is automatically assigned. Hyperparameter optimization was performed on 20% of the dataset, whereas the remaining set (80%, 388 records) was used to train and test the model. We also calculated the importance of features in predicting the targeted outcome by computing the mean impurity decrease in decision tree-based models (RF) after the training step.

Evaluation

To train and test the performance of the machine learning models, stratified 10-fold cross-validation was utilized. Cross-validation techniques are re-sampling techniques used to divide the dataset into training and testing (held-out) sets. The training sets were used to train the machine learning model, whereas the testing set was used to evaluate the model performance. We implemented a stratified cross-validation technique to ensure that each class was adequately represented in both the training and test sets. To evaluate the model performance, we used four metrics: sensitivity (true positive rate (TPR)), specificity (true negative rate (TNR)), overall accuracy, and F1 measure. Sensitivity and specificity were used to evaluate the model performance in discriminating between one class and the other. The sensitivity or TPR was calculated as the proportion of true-positive outcomes (correctly predicted as positive outcomes) among the total number of positive outcomes. Specificity or TNR is the proportion of true-negative outcomes (correctly assigned to the negative class) to the total number of negative examples.

The article "Machine Learning-Based Prediction of COVID-19 Prognosis Using Clinical and Hematologic Data" was retracted in 2026. Reasons: unreliable results or conclusions; concerns about the data; concerns about the methods; concerns about the results or conclusions.

Overall accuracy is the proportion of correctly classified instances (both positive and negative) among the total number of examined instances. In binary classification, accuracy is equal to the true positive (TP) added to the true negative (TN) divided by the total number of examples. The F1 measure is calculated as the harmonic mean of precision, which is the true positive example among all the predicted positive samples and sensitivity values. The area under the receiver operating characteristic (ROC) curve (AUC) is a discriminating performance indicator that indicates how well a model can distinguish between cases (positive instances) and non-cases (negative instances). We implemented machine learning models on a different set of features to predict the clinical outcomes and disease severity in infected patients. First, we examined the model performance on the entire set of features (45 attributes), including demographics, comorbidities, clinical and hematological attributes, and medications. We then examined each type of feature separately to assess their discriminative power in predicting COVID-19 outcome and severity.

## Results

Patients’ demographic characteristics

Table 1 and Table 2 present the patients’ clinical and hematological data. The study cohort comprised 485 patients with COVID-19, 116 women and 369 men, with an average of 45.36 years and a range between 18 and 90 years. Of these patients, 386 recovered and 99 died; 371 were not admitted to the ICU, and 114 were admitted to the ICU. All patient information was collected during their initial admission to the hospital, but medical treatment, clinical outcome, and disease severity information were obtained after admission to the hospital.

**Table 1:** Demographic and clinical data of the included patients

Character			Percentage (%)
Demographic data	Age Min=18, Max=90, Mean=45.36		
	Gender	Female	23.9%
		Male	76.1%
	Nationality	Saudi	23.1%
		Non-Saudi	76.9%
	Job	Healthcare worker	4.9%
		Non-healthcare worker	95.1%
Comorbidities	Diabetes		25.2%
	Hypertension		22.7%
	Respiratory		4.5%
	Malignancy		1.2%
	Cardiovascular		5.6%
Symptoms at admission	Fever		45.1%
	Cough		62.7%
	Dyspnea		29.7%
	Sore throat		22.3%
	Loss smell/taste		3.7%
	Gastrointestinal disturbance		15.7%
	Others		14.0%
Signs at lung X-ray/CT	Positive		67.2%
Medication during hospital admission	Paracetamol		100.0%
	Anticoagulants		13.0%
	Azithromycin		40.0%
	Other antibiotic		52.6%
	Oseltamivir		40.4%
	Kaletra		8.5%
	Hydroxychloroquine (HCQ)		21.2%

The article "Machine Learning-Based Prediction of COVID-19 Prognosis Using Clinical and Hematologic Data" was retracted in 2026. Reasons: unreliable results or conclusions; concerns about the data; concerns about the methods; concerns about the results or conclusions.

**Table 2:** Hematological data of included patients at admission

Parameter	Min	Max	Mean
Hemoglobin level (g/dL)	4.0	116	13.54
Red blood cells (M/uL)	1.37	13.8	4.89
White blood cells (K/uL)	1.53	35.1	7.66
Platelets (K/uL)	0.2	886	248.11
Basophils (%)	0.0	11.9	0.93
Neutrophil (%)	2.78	6201	78.77
Monocytes (%)	0.2	68	7.91
Lymphocytes (%)	0.0	73.9	24.48
Eosinophil (%)	0	42.3	1.34
Basophils (K/uL)	0.0	0.77	0.078
Neutrophils (K/uL)	0.2	32.2	5.46
Monocytes (K/uL)	0.1	17.9	0.71
Lymphocytes (K/uL)	0.0	28	1.55
Eosinophil (K/uL)	0.0	3.08	0.093
D-Dimer (mg/L)	0.092	100	3.176
Prothrombin time (seconds)	9.6	38.2	12.52
Activated partial thromboplastin time (aPTT) (seconds)	17.4	83.6	32.91
International normalised ratio (INR) (%)	0.7	4.1	1.10
Ferritin (ng/ml)	6.69	12606	784.53
C-reactive protein(mg/L)	0.41	273	45.42
Glucose (mg/dL)	82.8	469	124.85

Predictive factors for COVID-19 outcome

Table 3 presents the results of the different machine learning models for predicting COVID-19 patient outcomes (i.e.,, death; positive class or recovery). The results demonstrate the performance using a different set of features and different classification approaches. Classifiers provided comparable results for all sets of features, but overall, SVM, and RF yielded the highest accuracy, F1 score, specificity (TNR), and AUC. Among all the sets of features, hematological variables gave the highest performance with 0.95 AUC and 0.95 sensitivity, and 0.72 specificity using RF yielded the best overall performance on hematological features. Thus, no significant reduction was observed in model performance when only hematological variables were included.

**Table 3:** Outcome prediction performance using different machine learning models. Logistic regression (LR), multilayer perceptron (MLP), random forest (RF), support vector machine (SVM), naive Bayes (NB), and extreme gradient boosting (XGboost), with a different set of features, clinical data, hematological parameters, medication, and a combination of all set of features. TPR: true-positive rate, TNR: true-negative rate, AUC: area under the curve

Type of features	Model	Accuracy	F1	TPR	TNR	AUC
Comorbidities	LR	0.78	0.88	0.99	0.05	0.62
	MLP	0.78	0.87	0.98	0.05	0.63
	RF	0.76	0.86	0.95	0.08	0.65
	SVM	0.78	0.88	0.99	0.01	0.45
	NB	0.77	0.86	0.95	0.12	0.63
	XGboost	0.78	0.87	0.99	0.01	0.62
Symptomatic observations	LR	0.82	0.89	0.91	0.53	0.83
	MLP	0.83	0.89	0.9	0.59	0.83
	RF	0.8	0.88	0.93	0.35	0.82
	SVM	0.78	0.88	0.99	0.04	0.82
	NB	0.83	0.89	0.89	0.6	0.84
	XGboost	0.8	0.88	0.93	0.35	0.83
Hematological variables	LR	0.89	0.93	0.93	0.73	0.95
	MLP	0.9	0.94	0.94	0.78	0.94
	RF	0.9	0.94	0.95	0.72	0.95
	SVM	0.89	0.93	0.93	0.75	0.94
	NB	0.8	0.89	1	0.09	0.87
	XGboost	0.9	0.94	0.94	0.74	0.95
Medical treatments	LR	0.81	0.89	0.96	0.27	0.77
	MLP	0.82	0.89	0.96	0.32	0.79
	RF	0.85	0.9	0.93	0.56	0.82
	SVM	0.82	0.89	0.97	0.29	0.65
	NB	0.82	0.89	0.97	0.29	0.78
	XGboost	0.83	0.9	0.94	0.42	0.8
All features	LR	0.88	0.92	0.93	0.72	0.94
	MLP	0.89	0.93	0.92	0.81	0.95
	RF	0.9	0.94	0.95	0.71	0.96
	SVM	0.9	0.94	0.93	0.8	0.95
	NB	0.8	0.89	1	0.12	0.91
	XGboost	0.9	0.94	0.94	0.74	0.95

Figure 1 shows the AUC performance using multiple classifiers with different sets of features. As shown in Figure 2, only the performances of the NB models decreased by 4%, while the MLP, RF, and SVM decreased by 1%. Clinical and symptomatic variables showed a lower performance in predicting death/recovery outcomes, with the best overall performance of 0.84 AUC, 0.89 sensitivity, and 0.60 specificity yielded using the NB model. The results also showed that comorbidities and medical treatments during the hospital stay did not lead to a powerful predictive performance. Figure 3 and Figure 4 show the performance of all the machine learning models trained on comorbidities and symptoms. The results were considerably low and relatively close to the ROC curve "no skill" performance.

The article "Machine Learning-Based Prediction of COVID-19 Prognosis Using Clinical and Hematologic Data" was retracted in 2026. Reasons: unreliable results or conclusions; concerns about the data; concerns about the methods; concerns about the results or conclusions.

**Figure 1:** Area under the ROC curve of predicting COVID-19 patient outcome (left) and ICU admission (right) using all sets of features AUC: area under the curve, ROC: receiver operating characteristic, COVID-19: coronavirus disease 2019, ICU: intensive care unit, LR: logistic regression, MLP: multilayer perceptron, RF: random forest, SVM: support vector machine, NB: naïve Bayes, XGboost: extreme gradient boosting

**Figure 2:** Area under the ROC curve of predicting the outcome of COVID patient outcome (left) and ICU admission (right) using hematological features AUC: area under the curve, ROC: receiver operating characteristic, COVID-19: coronavirus disease 2019, ICU: intensive care unit, LR: logistic regression, MLP: multilayer perceptron, RF: random forest, SVM: support vector machine, NB: naïve Bayes, XGboost: extreme gradient boosting

**Figure 3:** Area under the ROC curve of predicting COVID patient outcome (left) and ICU admission (right) using clinical features. AUC: area under the curve, ROC: receiver operating characteristic, COVID-19: coronavirus disease 2019, ICU: intensive care unit, LR: logistic regression, MLP: multilayer perceptron, RF: random forest, SVM: support vector machine, NB: naïve Bayes, XGboost: extreme gradient boosting

**Figure 4:** Area under the ROC curve of predicting COVID patient outcome (left) and ICU admission (right) using comorbidities features. AUC: area under the curve, ROC: receiver operating characteristic, COVID-19: coronavirus disease 2019, ICU: intensive care unit, LR: logistic regression, MLP: multilayer perceptron, RF: random forest, SVM: support vector machine, NB: naïve Bayes, XGboost: extreme gradient boosting

Predictive factors for COVID-19 severity

The results of various machine learning models in predicting the severity of COVID-19 (i.e., ICU admission; positive class or no ICU admission) are presented in Table 4. The results showed that the complete set of patient features indicated the severity of the case. Models, in general, yielded a comparative performance, yet XGboost yielded the best overall performance. The XGboost model that is trained on all the features provided predictive accuracy, F1 score, sensitivity, specificity, and AUC of 0.92, 0.84, 0.79, 0.97, and 0.96, respectively. Hematological variables gave a very good performance in predicting disease severity, with the best overall performance of 0.92 accuracy, 0.83 F1 score, 0.78 sensitivity, 0.97 specificity, and 0.95 AUC yielded using the XGboost classifier. Machine learning models trained on comorbidities exhibited very low performance compared with other sets of features. However, medical treatments during hospital stay provided better predictive performance, as shown in Figure 3 and Figure 5.

The article "Machine Learning-Based Prediction of COVID-19 Prognosis Using Clinical and Hematologic Data" was retracted in 2026. Reasons: unreliable results or conclusions; concerns about the data; concerns about the methods; concerns about the results or conclusions.

**Table 4:** ICU admission prediction performance using different machine learning models Logistic regression (LR), multilayer perceptron (MLP), random forest (RF), support vector machine (SVM), naive Bayes (NB), and extreme gradient boosting (XGboost), with a different set of features. FPR: false-positive rate, TPR: true-positive rate, TNR: true-negative rate, AUC: area under the curve

Type of Features	Model	Accuracy	F1	FPR	TPR	AUC
Comorbidities	LR	0.74	0.17	0.1	0.96	0.62
	MLP	0.7	0.18	0.11	0.96	0.63
	RF	0.74	0.14	0.08	0.96	0.61
	SVM	0.74	0	0	1	0.55
	NB	0.73	0.17	0.11	0.94	0.64
	XGboost	0.74	0.14	0.08	0.97	0.61
Symptomatic observations	LR	0.84	0.67	0.66	0.9	0.85
	MLP	0.84	0.67	0.64	0.91	0.85
	RF	0.82	0.63	0.6	0.9	0.84
	SVM	0.82	0.66	0.68	0.87	0.84
	NB	0.84	0.68	0.67	0.9	0.84
	XGboost	0.8	0.65	0.62	0.91	0.85
Hematological variables	LR	0.9	0.8	0.77	0.94	0.95
	MLP	0.9	0.8	0.82	0.92	0.95
	RF	0.9	0.8	0.73	0.97	0.95
	SVM	0.91	0.81	0.77	0.96	0.95
	NB	0.77	0.17	0.09	1	0.89
	XGboost	0.92	0.83	0.78	0.97	0.95
Medical treatments	LR	0.81	0.52	0.39	0.96	0.78
	MLP	0.86	0.67	0.58	0.96	0.8
	RF	0.86	0.69	0.62	0.94	0.82
	SVM	0.81	0.45	0.3	0.98	0.68
	NB	0.81	0.45	0.3	0.98	0.78
	XGboost	0.86	0.67	0.58	0.96	0.82
All features	LR	0.9	0.81	0.81	0.93	0.96
	MLP	0.91	0.81	0.82	0.93	0.96
	RF	0.91	0.81	0.75	0.97	0.96
	SVM	0.91	0.82	0.79	0.95	0.96
	NB	0.79	0.28	0.16	1	0.92
	XGboost	0.92	0.84	0.79	0.97	0.96

The article "Machine Learning-Based Prediction of COVID-19 Prognosis Using Clinical and Hematologic Data" was retracted in 2026. Reasons: unreliable results or conclusions; concerns about the data; concerns about the methods; concerns about the results or conclusions.

**Figure 5:** Area under the ROC curve of predicting COVID patient outcome (left) and ICU admission (right) using medical treatments features AUC: area under the curve, ROC: receiver operating characteristic, COVID-19: coronavirus disease 2019, ICU: intensive care unit, LR: logistic regression, MLP: multilayer perceptron, RF: random forest, SVM: support vector machine, NB: naïve Bayes, XGboost: extreme gradient boosting

To measure feature importance, we analyzed the mean decrease in impurity in the RF model after training on a different set of features. The results showed that among the 45 features, the most influential features in predicting patient outcome were hematological variables predicting patient outcome and disease severity (see Figure 6). Furthermore, among the hematological variables, we found that the most important features were neutrophils, D-dimer, lymphocytes, and monocytes for predicting both ICU admission and patient outcome.

**Figure 6:** Hematology variables feature importance in predicting patient outcome (left) and ICU admission (right). WBC: white blood cells, APTT: activated partial thromboplastin time, INR: international normalized ratio, Hb: hemoglobin, RBC: red blood cells, CT: computed tomography

## Discussion

Recently, utilizing machine learning in medicine has become of great interest in fostering clinical research and predicting the diagnosis and prognosis of many diseases [7]. Our research group previously confirmed the efficacy of using machine learning models to predict the diagnosis of COVID-19 [4]. The accuracies were 82% and 81% for diagnosing COVID-19 using NB and LR, respectively. The most significant features for predicting COVID-19 diagnosis at admission were basophil count, lung radiography, eosinophil count, and loss of smell. In the current study, we aimed to explore the feasibility of predicting COVID-19 outcome and severity based on hematological and clinical data using machine learning techniques.

The results of the current study emphasize the importance of patients’ hematological parameters at admission in the prediction of both COVID-19 outcome and severity. Among all the tested hematological parameters, neutrophils and lymphocytes were the most important features in predicting both COVID-19 outcome and severity in our population. This finding is consistent with recent studies that supported the association between lymphocytes and COVID-19 severity [10,11]. However, the models from both studies provided lower sensitivity, specificity, and accuracy for predicting COVID-19 severity than our model. Several previous clinical studies have reported an association between the neutrophil-to-lymphocyte ratio (NLR) and COVID-19 severity and outcome [12,13]. In addition, NLR has been studied as a prognostic predictive factor for other infections [8]. Furthermore, the dynamic relationship between neutrophils and viral infections has been emphasized and investigated in-depth, as well as the impact of neutrophils on cytokine storms and COVID-19 severity [14]. Similarly, D-dimer was the third most important feature to predict COVID-19 death and the second most important predictor of ICU admission. This finding is consistent with that of a previous study [15] showing that D-dimer was the second most important feature in machine learning models to predict ICU admission and ventilation risk in the Los Angeles population. Moreover, this is aligned with previously reported clinical studies that support the association between D-dimer levels and thromboembolism events with poor COVID-19 prognosis [16,17]. 

The article "Machine Learning-Based Prediction of COVID-19 Prognosis Using Clinical and Hematologic Data" was retracted in 2026. Reasons: unreliable results or conclusions; concerns about the data; concerns about the methods; concerns about the results or conclusions.

Remarkably, the results of the current study showed that the clinical manifestations at admission had a lower performance in predicting COVID-19 outcome and severity. This result was expected, as COVID-19 has symptoms similar to several other viral respiratory infections [18]. By contrast, previous research has shown that anosmia and olfactory dysfunctions are good prognostic factors [19]. The discrepancy between that study and the current one could be explained by the fact that our study participants were hospitalized patients; however, anosmia is associated with mild COVID-19 cases. Indeed, the percentage of COVID-19 patients who reported anosmia in our study was relatively low. By contrast, another machine learning study showed that anosmia is a good predictor for diagnosing new COVID-19 cases with 82% sensitivity, 78% specificity, and 80% accuracy [20].

The current study showed that medical treatment during admission was a better predictor of ICU admission than the risk of death. However, these interesting findings must be interpreted carefully, and more studies must be conducted to further analyze the impact of different treatment doses, durations, and regimens on COVID-19 prognosis. Unexpectedly, the results from the current study showed that comorbidities were poor predictors of COVID-19 outcome and severity. However, the results of a meta-analysis regarding the effect of comorbidities on COVID-19 prognosis are controversial. Previous meta-analysis showed that comorbidities are associated with an increased risk of ICU admission and death [21], while another meta-analysis rejected this association [22]. This discrepancy was argued by another meta-analysis that revealed that geographic location contributes to the association between comorbidities and COVID-19 prognosis [23].

The article "Machine Learning-Based Prediction of COVID-19 Prognosis Using Clinical and Hematologic Data" was retracted in 2026. Reasons: unreliable results or conclusions; concerns about the data; concerns about the methods; concerns about the results or conclusions.

This study, despite its significant contributions, has some limitations. First, it relied on retrospective data, which can introduce bias and confounders. The study also used a relatively small sample size. Furthermore, the data used in the study were collected during the peak of the pandemic, which may not reflect the current situation, especially with the introduction of new variants and advancements in treatments. Finally, the study was based on data from a single country, Saudi Arabia, which limits its generalizability to other global contexts.

## Conclusions

Neutrophils, lymphocytes, and D-dimer levels were the most significant predictive features in our population. Therefore, the results of this study can be effectively utilized to predict the severity and outcome of COVID-19 patients and improve patient healthcare. Despite the important finding in the current study, the relatively small sample size may limit its clinical application. Moreover, the retrospective nature of the study was one of the limitations. Thus, the results from this study must be compared with those of ongoing COVID-19 clinical trials to verify the accuracy of our prediction model.

Moreover, in this study several machine learning models were implemented with a different set of features including clinical, hematological, medication, comorbidities, and medications variables to predict the severity and outcomes of COVID-19. The results show variabilities in the performance according to the used features with hematological variables demonstrating superior predictive capabilities compared to other feature sets.

Our investigation revealed that the performance of the machine learning models was subject to variability depending on the chosen methodology, with XGboost, MLP, and RF emerging as consistently outperforming models in predicting outcomes in our analyses. These observed variations underscore the nuanced influence of both feature selection and model choice on the predictive accuracy of our models, providing valuable insights for future research and clinical applications.
